The article "Increased Rotatory Laxity after Anterolateral Ligament Lesion in Anterior Cruciate Ligament- (ACL-) Deficient Knees: A Cadaveric Study with Noninvasive Inertial Sensors" was published in 2021. Journal: Biomed Res Int.

# Increased Rotatory Laxity after Anterolateral Ligament Lesion in Anterior Cruciate Ligament- (ACL-) Deficient Knees: A Cadaveric Study with Noninvasive Inertial Sensors

**DOI:** 10.1155/2021/7549750

**Published:** 2021-07-06

**Authors:** Alberto Grassi, Tommaso Roberti di Sarsina, Stefano Di Paolo, Cecilia Signorelli, Tommaso Bonanzinga, Federico Raggi, Massimiliano Mosca, Stefano Zaffagnini

**Affiliations:** ^1^Clinica Ortopedica e Traumatologica II, IRCCS Istituto Ortopedico Rizzoli, Bologna 40136, Italy; ^2^Dipartimento di Scienze Biomediche e Neuromotorie, Università di Bologna, Bologna 40136, Italy; ^3^Centro per la Ricostruzione Articolare del Ginocchio, Humanitas Research Hospital, Rozzano MI, Italy

## Abstract

The anterolateral ligament (ALL) has been suggested as an important secondary knee restrain on the dynamic laxity in anterior cruciate ligament- (ACL-) deficient knees. Nevertheless, its kinematical contribution to the pivot-shift (PS) phenomenon has not been clearly and objectively defined, and noninvasive sensor technology could give a crucial contribution in this direction. The aim of the present study was to quantify in vitro the PS phenomenon in order to investigate the differences between an ACL-deficient knee and an ACL+ALL-deficient knee. Ten fresh-frozen paired human cadaveric knees (*n* = 20) were included in this controlled laboratory study. Intact, ACL-deficient, and ACL+ALL-deficient knees were subjected to a manual PS test quantified by a noninvasive triaxial accelerometer (KiRA, OrthoKey). Kinematic data (i.e., posterior acceleration of the tibial lateral compartment) were recorded and compared among the three statuses. Pairwise Student's *t*-test was used to compare the single groups (*p* < 0.05). Intact knees, ACL-deficient knees, and ACL+ALL-deficient knees showed an acceleration of 5.3 ± 2.1 m/s^2^, 6.3 ± 2.3 m/s^2^, and 7.8 ± 2.1 m/s^2^, respectively. Combined sectioning of ACL and ALL resulted in a statistically significant acceleration increase compared to both the intact state (*p* < 0.01) and the ACL-deficient state (*p* < 0.01). The acceleration increase determined by isolated ACL resection compared to the intact state was not statistically significant (*p* > 0.05). The ALL sectioning increased the rotatory laxity during the PS after ACL sectioning as measured through a user-friendly, noninvasive triaxial accelerometer.

## 1. Introduction

The pivot-shift (PS) phenomenon has been described as anterior subluxation of the lateral tibial plateau followed by its sudden reduction during combined stresses [1]. Specifically, the pivot-shift test has been defined as a combination of valgus stress and internal tibial rotation during limb flexion [2]. This phenomenon has been widely identified as one of the essential signs of functional anterior cruciate ligament (ACL) insufficiency [2, 3]. Moreover, literature reports that the grade of pivot-shift correlates more closely with patient satisfaction and symptoms of functional instability than Lachman and drawer tests that address only static joint laxity [4]. Since the pivot-shift phenomenon has been associated with dynamic instability of the joint [1], clinicians have been trying to recreate this abnormality by applying combined stresses to the limb to highlight its presence. Clinical and basic research on the PS test has increased over the past decade [5], and the importance of the secondary restraints of the knee emphasized [6], suggesting the anterolateral ligament (ALL) as an important restrain to control rotational laxity [7].

While there have been recent developments in understanding the incidence and anatomy of the ALL, its kinematic role and clinical relevance are yet to be fully determined. Some studies quantifying the contribution of the anterolateral capsule and the ALL to a simulated pivot-shift test in an in vitro setting suggested that the ALL acts as an effective secondary stabilizer throughout flexion when an internal rotation torque is applied in ACL-deficient knees [8, 9]. However, the instruments employed up to now, such as electromagnetic sensors [5, 10], robotic systems, and navigation systems [11, 12], are generally invasive, time-consuming, and expensive to be practical for routine use besides research purposes [13–15]. To overcome the latter issues, user-friendly and noninvasive devices based on triaxial accelerometer technology, e.g., the KiRA (OrthoKey, Lewes, DE, USA), were developed and validated for the quantitative assessment of rotatory knee laxity [16]. Such devices can be used in everyday clinical practice either in the operative room for underanesthesia evaluation or during clinical consultation for diagnosis and follow-up controls. In the context of combined ALL and ACL tears, an accurate assessment of the rotatory knee laxity by means of such devices might provide a valid support to the clinicians in the choice of surgical and postsurgical procedures.

Therefore, the aim of this study was to investigate in a cadaveric setting the effect of ALL sectioning on the dynamic laxity parameters of the ACL-deficient knee using noninvasive skin fixed inertial sensors. The hypothesis was that ALL sectioning would increase rotatory laxity measured with an inertial sensor during the PS after ACL sectioning.

## 2. Materials and Methods

### 2.1. Specimen Demographics and Preparation

All the biomechanical tests have been performed at Laboratorie d'Anatomie, Universitè Françoise-Rabelais. The study received IRB approval (Prot. 0006323 of 22/02/2013).

Ten fresh-frozen paired human cadaveric knees (all male, mean age 79, range 74-84 years old) with no prior injury, knee surgery, or gross anatomical abnormalities were included in the present study (*n* = 20). All specimens (full-legs) were stored at -20°C and thawed at room temperature for at least 36 hours before the testing session. The skin and the subcutaneous fatty tissue within 15 cm from the joint line on the tibia, fibula, and femur were removed to expose the ligamentous and tendinous structures that were left intact.

A medial parapatellar arthrotomy was performed to assess the knee joint status and allow access to the ACL. After separating the iliotibial tract fibers, a manual internal torque at 90° of flexion was applied to identify the ALL (Figure 1). The ALL was identified as the fanlike group of fibers originating from a point proximal and posterior to the Lateral Collateral Ligament (LCL) and inserted midway between the fibular head and Gerdy's tubercle; these fibers had an oblique course and tightened during internal knee rotation. The ALL was isolated from the capsule in each specimen. The PS test was then performed and evaluated by a noninvasive inertial sensor (intact status). Then, the ACL was resected from the femoral side through the open arthrotomy (ACL status). This was done to ensure the full ligament release from the femur and avoid the damage of lateral meniscus insertions. Lastly, the ALL was also resected, and the laxity test was repeated (ACL+ALL status). The ALL was sectioned last to assess its secondary role in controlling knee joint stability in the context of an ACL tear.

### 2.2. Setup

Knee dynamic laxity was evaluated with a noninvasive skin-fixed inertial sensor. Such device integrates a triaxial accelerometer (12 bit, ±8 g range) and a triaxial gyroscope (16 bit, ±2000 dpm range), wirelessly connected to a laptop for processing the acquired data (Figure 2).

The sensors were securely fixed on the skin through the masking tape between the lateral aspect of the anterior tuberosity and Gerdy's tubercle to achieve optimal stability and to minimize skin artifacts during the PS maneuver (Figure 3). The sensor position was chosen to detect the acceleration of the lateral tibial compartment, which is the most reliable in predicting high-grade PS phenomenon [17]. The main axis of the sensor was aligned with the tibial mechanical axis.

### 2.3. Dynamic Laxity Testing

A single surgeon, an expert in biomechanical testing, performed the ligament cutting and the laxity examination.

Intact, ACL-deficient, and ACL+ALL-deficient cadaveric knees were subjected to the PS test performed manually in the way described in the literature [1–3], using the standardized maneuver as reported by Hoshino et al. [18, 19]. Three test repetitions per condition were performed.

Between the analysis of each testing status, the specimen was maintained damp, applying a saline solution.

The repeatability of the PS test during manual-maximum execution has been thoroughly analyzed in a previous study using both the navigation system [20] and the inertial sensors [16].

### 2.4. Data Collection and Statistical Analysis

Normal distribution was verified by the Kolmogorov-Smirnov test. Three tested statuses were analyzed: intact, ACL-deficient, and ACL+ALL-deficient knees. One-way ANOVA was used to compare the three conditions. Pairwise comparisons were performed through Student's *t*-test with Dunn-Sidak *p* value adjustment for multiple comparisons. Differences between groups were considered statistically significant for *p* < 0.05.

An a priori power analysis was performed in order to identify an adequate sample size. Based on an alpha level of 0.05, a minimum of 10 specimens was required to detect statistical differences with an ES = 1.0 (large) and 80% power.

All the statistical analyses were computed in MATLAB (The MathWorks, Inc., Natick, Massachusetts, USA).

## 3. Results

The Kolmogorov-Smirnov test confirmed the normal distribution of all the acquired data, and it was possible to use parametric statistical tests. Therefore, the results for the intact, ACL-deficient, and ACL+ALL-deficient statuses were reported as mean ± SD.

A statistically significant difference (*p* < 0.001) was found among the three groups. The mean acceleration detected with the inertial sensor during the PS was 5.3 ± 2.1 m/s^2^ in the intact status, 6.3 ± 2.3 m/s^2^ after isolated ACL sectioning, and 7.8 ± 2.1 m/s^2^ after combined ACL+ALL sectioning (Table 1).

An increased acceleration of 1.0 ± 1.1 m/s^2^ was found between intact and ACL statuses; this difference was not significant.

A statistically significant (*p* < 0.001) difference of 1.5 ± 1.3 m/s^2^ was found between ACL and ACL+ALL statuses. Lastly, the overall difference between intact status and ACL+ALL status was 2.5 ± 1.3 m/s^2^ (*p* < 0.001) (Table 2).

## 4. Discussion

The most important finding of the present study was that sectioning the ALL leads to increased PS acceleration in the context of ACL-deficient knee as measured with a user-friendly noninvasive accelerometer (KiRA device). The latter device could be therefore proposed as an accurate and valid alternative to the gold standard for the quantitative assessment of rotatory knee laxity.

A combined injury to the ACL and ALL resulted in a significant increase in acceleration compared to the isolated ACL tear and the intact state. The increase in acceleration determined by the isolated ACL resection was not statistically significant, although showing a higher acceleration than the intact state. Similar findings were reported by Monaco et al. [21] in a comparable cadaveric setup. The authors sequentially sectioned the ACL and the whole anterolateral capsule and reported an increase of PS grade only after sectioning both the two structures, but not after isolate ACL removal. However, the authors evaluated rotatory laxity only with manual testing and without specific devices. More recent studies performed a similar investigation using specific robots for simulated pivot-shift evaluation. Spencer et al. [22] assessed the biomechanical function of the ALL during a simulated PS and reported an increase of the internal rotation during the early phase of the test. Through a similar setting, Rasmussen et al. [8] found a significant increase in axial plane translation in ACL+ALL-deficient knees when compared to isolated ACL sectioning at 0°, 15°, 30°, and 60° of flexion. Yasuma et al. also reported an increased knee rotatory laxity in six fresh-frozen cadavers in the presence of anterolateral structure tears [23]. On the other hand, other authors [24–29] that compared the effect of an isolated ALL and iliotibial band resection in an ACL-intact knee did not report significant correlations with tibiofemoral compartment subluxation during a simulated pivot-shift, thus suggesting that the ALL does not represent a primary restraint to the pivot-shift test. The heterogeneous results might be due to the different setups adopted, the age of the specimens and relative quality of the knee structures, and the instrumented device used for the quantitative assessment.

From a clinical perspective, the results of the present study are consistent with those obtained by Muccioli et al. [30]. The authors tested the KiRA device in vivo on 60 ACL-injured patients and reported an average side-to-side difference of 0.8 m/s^2^ between knees with “glide” PS and contralateral healthy knee. The latter results are comparable with the difference of 1.0 m/s^2^ reported between intact and ACL groups in the present study. Similarly, the difference of 2.9 m/s^2^ reported by Muccioli et al. [30] between knees with “gross” PS and healthy contralateral side is comparable to 2.5 m/s^2^ found between intact and ACL+ALL statuses.

Also, a previous international, multicenter prospective cohort study [31] tested the KiRA device. In a more complex evaluation, the multiple examiners used the same standardized technique to perform the PS, finding a significant positive association between the clinical PS graded according to the IKDC score and quantitative measures of tibial acceleration of this noninvasive device over a cohort of 103 patients with an ACL injury. In their study, patients with associated lesions were included to collect a wider ACL injured population with high- and low-grade pivot-shift test results.

To the best of our knowledge, no previous studies quantitatively investigated the effect of the ALL on knee laxity with noninvasive technologies. The capability of the KiRA accelerometer to detect different grades of pivot-shift opens the possibility of identifying patients with an unrecognized associated lesion. Based on these considerations, it could be suggested that the KiRA accelerometer sensor could be helpful to objectively define high-grade PS and possibly assist the clinician in diagnosing ALL injury. Such investigation could indeed be conducted pre-, intra-, and postoperatively without the need of invasive devices like the surgical navigation system.

The authors noted some limitations. First, the sample size was small, and the age of the specimens was not similar to the typical ACL-injured population; however, these are common drawbacks of in vitro kinematic studies. Second, the KiRA accelerometer has lower accuracy compared to robot systems used in similar in vitro investigations [32]. However, the device could detect changes of the PS, achieving results comparable to similar studies using robotic systems. Third, joint acceleration is the only parameter measurable through the KiRA device. However, it has been proved that joint acceleration significantly correlates rotatory laxity with patients' clinical perception of joint instability. Last, although high repeatability had already been demonstrated for the current device [16], the examiner conducted both the cuts and the laxity tests and was not blind for the status of the knee.

## 5. Conclusion

The ALL sectioning increased the rotatory laxity during the PS after ACL sectioning as measured through a user-friendly noninvasive triaxial accelerometer. The KiRA triaxial accelerometer could be proposed as a noninvasive and user-friendly tool to assist clinicians in diagnosing combined ACL and ALL injuries and quantifying the rotational laxity.

## Figures and Tables

**Figure 1:** Detail of the knee anterolateral ligament. GT = Gerdy's tubercle; LE = lateral epicondyle; LM = lateral meniscus; FH = fibula head.

**Figure 2:** The KiRA triaxial accelerometers for noninvasive quantitative assessment of rotatory laxity. On the left, the representation of sensor placement with respect to the tibial mechanical axis; on the right, a typical pivot-shift acceleration chart visualized real-time in the KiRA software environment.

**Figure 3:** Examination setting. (a) Detail of structures under investigation after skin and fatty tissue removal; (b) full-leg view with the examiner (in white, the accelerometer secured to the skin).

**Table 1:** Pivot-shift dynamic laxity assessment in the different knee statuses through the KiRA device.

	Intact	ACL deficient	ACL+ALL deficient	*p* value
PS acceleration (m/s^2^)	5.3 ± 2.1	6.3 ± 2.3	7.8 ± 2.1	<0.001^∗^

Note: ACL: anterior cruciate ligament; PS: pivot-shift; ALL: anterolateral ligament; asterisk represents statistically significant differences (ANOVA); data are expressed as mean ± standard deviation.

**Table 2:** Multiple comparisons between the pivot-shift accelerations in the different knee statuses.

	Diff (m/s^2^)	*p* value
Intact vs. ACL deficient	1.0 ± 1.1	0.06
Intact vs. ACL+ALL deficient	2.5 ± 1.3	<0.001^∗^
ACL vs. ACL+ALL deficient	1.5 ± 1.3	<0.001^∗^

Note: ACL: anterior cruciate ligament; PS: pivot-shift; ALL: anterolateral ligament; asterisk represents statistically significant differences (Student's *t*-test with Dunn-Sidak correction); data are expressed as mean ± standard deviation.

## Data Availability

Data are available on reasonable request.
